The article "Effects of Bacillus subtilis as a single strain probiotic on growth, disease resistance and immune response of striped catfish (Pangasius hypophthalmus)" was published in 2024. Journal: PLoS One.

# Effects of *Bacillus subtilis* as a single strain probiotic on growth, disease resistance and immune response of striped catfish (*Pangasius hypophthalmus*)

**DOI:** 10.1371/journal.pone.0294949

**Published:** 2024-01-30

**Authors:** Razia Liaqat, Shafaq Fatima, Wajeeha Komal, Qandeel Minahal, Zakia Kanwal, Muhammad Suleman, Chris G. Carter

**Affiliations:** 1 Department of Zoology, Lahore College for Women University, Lahore, Punjab, Pakistan; 2 Department of Biological Sciences, Purdue University Fort Wayne, Fort Wayne, IN, United States of America; 3 Institute of Microbiology, University of Veterinary and Animal Sciences Lahore, Lahore, Pakistan; 4 Aquaculture Nutrition at the Institute for Marine and Antarctic Studies (IMAS), University of Tasmania, Hobart, Australia; Tanta University Faculty of Agriculture, EGYPT

## Abstract

The present study investigated the potential role of *Bacillus subtilis* as probiotic in striped catfish (*Pangasius hypophthalmus*). Fish (initial weight = 150.00±2.63g n = 180) were stocked in circular tanks. Four isonitrogenous (30%) and isolipidic (3.29%) diets were formulated having supplementation of *B*. *subtilis* at four different levels (P0; 0, P1: 1×10^6^, P2: 1×10^8^ and P3: 1×10^10^ CFU/g). Each treatment had three replicates, while each replicate had fifteen fish. The trial started on second week of July and continued for eight weeks. Growth, feed conversion ratio, crude protein content, the concentration of amylase and protease, the profile of both dispensable and non-dispensable amino acids in all four dietary groups increased with a gradual increase of *B*. *subtilis* in the diet. At the end of growth experiment, fish in all four groups were exposed to *Staphylococcus aureus* (5×10^5^ CFU/ml). After *S*. *aureus* challenge, fish fed with *B*. *subtilis* responded better to damage caused by reactive oxygen species and lipid peroxidation and better survival rate. The catalase and superoxide dismutase level also increased in response to bacterial challenge in *B*. *subtilis* fed groups. On the other hand, the concentration of malondialdehyde gradually decreased in these groups (+ve P0 >P1>P2>P3). It is concluded that supplementation of *B*. *subtilis* as a probiotic improved the growth, protein content, antioxidant response and immunocompetency against *S*. *aureus* in striped catfish. The optimum dosage of *B*. *subtilis*, at a concentration of 1×10^10^ CFU/g, resulted in the most favorable outcomes in striped catfish. This single bacterial strain can be used as an effective probiotic in large scale production of aquafeed for striped catfish. Future studies can investigate this probiotic’s impact in the intensive culture of the same species.

## 1. Introduction

The Striped catfish (*Pangasius hypophthalmus*) is widely recognized as an exceptional aquaculture species which is ideally suited for warm climates. It occupies a prominent position as a primary aquaculture commodity in international markets, holding the status of the second most produced prominent species, surpassed only by tilapia [1]. The global production of striped catfish was recorded as 2520.41 thousand tons in 2022 [2]. In South Asia, aquaculture is a rapidly expanding industry; therefore, species diversification is an indispensable measure for the advancement and sustainability of this sector. One of the finest opportunities to stimulate investment and foster the expansion of aquaculture in South Asia is the cultivation of striped catfish. This species flaunts a proven breeding, husbandry protocols, and already possesses an established market, making it an ideal choice [1]. However, ensuring sufficient nutrition becomes paramount for augmenting striped catfish production since it constitutes 40–50% of the cumulative production expenditure [3]. In intensive aquaculture, it is possible to provide fish with a diet of superior quality and adequately balanced [4]. Moreover, it facilitates the cultivation of fish with high stocking biomass, necessitating minimal investment yet generating enhanced profitability [5]. However, the rate of pathogen transmission could be heightened through increased stocking biomass [6]. In fact, intensive farming environments are considered evolutionary hotspots, wherein the escalated transmission and frequency of infections could promote virulence in pathogen populations [7, 8].

In recent decades, intensive systems of striped catfish have suffered substantial economic losses (US $60 million annually) due to disease outbreaks by pathogenic organisms [9, 10]. More than 92 genera of pathogens are responsible for this economic loss including, *Aeromonas* (60–70%), *Staphylococcus* (70%), *Pseudomonas* (50%), *Edwardsiella ictaluri* (50–70%), *Shigella* (32%) and *Salmonella* (3.22%) [11–13]. Among the various species of freshwater and marine fish, *S*. *aureus*, is recognized as one of the most commonly encountered pathogens, with a prevalence rate of 40–60% in fish farming and an astonishing 87% in associated products [14, 15]. Fish handlers are the common vectors of this bacterium, transmitting the infection to fish at the stage of stocking, feeding, harvesting, and processing e.g., approximately 30% of exported striped catfish fillets to Poland were found to be contaminated with coagulase-positive *Staphylococcus aureus* [16].

To mitigate the risk posed by all pathogens, a range of antibiotics, pesticide residues, and chemical products have been employed [17]. However, the excessive and unjustified use of antibacterials for pathogen prevention and growth stimulation has led to the emergence of antibiotic resistance. Nonetheless, instead of relying on antibiotics, several ecologically sustainable biological approaches have been developed, emphasizing the significance of probiotic administration as a central focus of aquaculture research [18, 19]. When administered in appropriate mixture and dose, probiotic bacteria are beneficial microorganisms that exert therapeutic effects in several species such as tilapia [20, 21], grass carp [17], and goldfish [22]. The effectiveness of probiotics in the aquaculture industry, including economic expansion, disease resistance (*Bacillus subtilis*- 60–70%) and high yield (*Bacillus licheniformis*—50%) has been conclusively illustrated [23, 24].

Probiotics empower fish to combat inherent stressors by reducing the quantities of reactive oxygen species (ROS) which are naturally produced during regular metabolic activities [25]. ROS commonly act as redox messengers determining cellular fate, and acting as signaling molecules for oxidative stress [26]. At low levels, antioxidant system can eliminate ROS. Nevertheless, when exposed to intense stimuli such as hypoxia, the excessive buildup of ROS disrupts the equilibrium within cells, resulting in oxidative stress and impairments in cellular functionality [27, 28]. Probiotic strains, such as *Bifidobacterium animalis*, *Lactobacillus rhamnosus*, and *Bacillus* spp. have exhibited substantial antioxidant potential and capabilities to alleviate oxidative damage [29, 30]. The potential mechanism underlying the antioxidant effects of probiotics encompass the autonomous secretion of antioxidant metabolites, adjustment of antioxidative activities, and suppression of enzyme activities implicated in the generation of ROS [31].

However, among all other probiotics, *Bacillus subtilis* is widely accepted in aquaculture due to its spore-forming ability [32], production of a broad spectrum of antibacterial substances [33], and the presence of high-antioxidant-activity substances such as superoxide dismutase (SOD) and glutathione (GSH) [34, 35]. Multiple studies substantiate the probiotic effects of *B*. *subtilis*, including the prevention of gastrointestinal disorders, leading to the improvement of pond water quality and the increased survival rate of animals in aquaculture [17, 36]. A study conducted by [37] examined the synergistic effects of *Bacillus* strains on the growth and immune response of striped catfish. However, to the best of our knowledge, the specific impact of a single strain, *B*. *subtilis*, has yet to be investigated in this species. The effectiveness of single strains was found to be comparable to that of multi-strains combinations. Single strain probiotic *B*. *subtilis* enhances survival rate (65–70%) [34], increases weight gain (50%) [38], improves digestive activity ([33], mitigates enteric septicemia in catfish (70–80%) [39], control *Aeromonas* infection in *Oreochromis mykiss* [40] and increases innate immunity and intestinal microbial population [41]. Therefore, the present investigation aims to study the potential effects of dietary supplementation of *B*. *subtilis* on growth efficiency, digestive enzyme activity, antioxidant mechanism, and immunological response in striped catfish.

## 2. Materials and methods

### 2.1 Preparation of experimental diets

In this study, commercial probiotic (ECOSH, Estonian) was used as a source of *B*. *subtilis*, contained a concentration of 1×10^12^ billion colony forming unit (CFU). One gram of probiotic containing 1×10^12^ billion CFU was used to obtained, final concentrations of 1×10^10^, 1×10^8^, and 1×10^6^ billion CFU of *B*. *subtilis*, respectively. The volume of desired probiotics was calculated, using following formulae and then mix with sterile distilled water.

Volumeofprobiotic=TargetCFU÷InitialCFU×Initialvolume

For confirmation of CFU in each concentration, plate count assay was performed using nutrient agar plate (HiMedia Ltd., Lahore, Pakistan). Plates were incubated for 24 hours at 37°C and number of colonies was counted afterwards by using a digital colony counter (Model: AVI-35). Treatment diets were prepared by mixing the finely ground ingredients (grains were procured from local farmers in Pakistan while origin of soybean was USA) (Table 1) with four levels of probiotics (P0: 0, P1: 1×10^6^, P2: 1×10^8^, P3: 1×10^10^CFU/g of the *B*. *subtilis* and pellets (1 mm) were prepared using pellet machine (PCSIR, Pakistan). The pellets were air-dried at room temperature and stored at 4°C. The treatment diets were formulated weekly to ensure the preservation of the actual bacterial count. Bacterial count in feed was performed after every three days using above mentioned plate count assay.

**Table 1:** Feed ingredients and chemical composition of experimental feed.

Ingredients (%)	P0 Diet	P1 Diet	P2 Diet	P3 Diet
Corn meal	28.00	28.00	28.00	28.00
Rice polish	12.00	12.00	12.00	12.00
Wheat bran	8.00	8.00	8.00	8.00
Canola meal	7.00	7.00	7.00	7.00
Soybean meal	36.00	36.00	36.00	36.00
APC	3.00	3.00	3.00	3.00
Dicalcium phosphate	3.00	3.00	3.00	3.00
Methionine	0.49	0.49	0.49	0.49
Lysine	1.32	1.32	1.32	1.32
L-Threonine	0.89	0.89	0.89	0.89
Axtra® XAP	0.15	0.15	0.15	0.15
MicroTech 40%	0.15	0.15	0.15	0.15
*B*.*subtilis* (CFU/g)	0	1×10^6^	1×10^8^	1×10^10^
**Chemical Composition of Feed**				
Moisture (%)	10.02	10.12	10.20	10.03
Crude Protein (%)	30.00	30.00	30.00	30.00
Crude Fat (%)	3.29	3.29	3.29	3.29
Crude Ash (%)	8.72	8.81	8.61	8.90

### 2.2 Growth experiment

Trial was started after ethical approval from Animal Ethics Committee (Zoo/LCWU/932). Fish were collected from a local hatchery and transported to the aquaculture facility at Lahore College for Women University. We acclimatized the fish in 600L tanks for a week. During acclimatization, the fish were fed with prepared feed without probiotics. After acclimatization, fish (initial weight = 150.00±2.63g n = 180) were stocked in 12 circular tanks (1.26 m^3^). Each treatment had three replicates, while each replicate had fifteen fish. An additional thirty fish were fed with a diet without probiotic to be used as the negative control in the bacterial challenge trial. These fish were reared in 2 separate circular tanks, (15 fish each) under the same husbandry conditions as other fish. The fish in each treatment group were fed three times a day. A total of 10% water in tank was exchanged on daily basis. Daily ration was calculated based upon 2% of biomass in that treatment group. The water quality parameters including dissolved oxygen (DO) (7.51±0.21mg/L), pH (7.21±0.41) and temperature (29.00±1.00°C) were monitored on a daily basis.

### 2.3 Sample collection

At the end of the growth experiment, fish were fasted for 24 hours and anesthetized using clove oil (Sigma Aldrich USA) (6ml/L). Five fish were randomly collected from each replicate of each treatment group. Total body weight and total body length, specific growth rate (SGR), feed conversion ratio (FCR), and weight of viscera, and liver were measured to calculate following parameters:

$$\text{Specific}\;\text{growth}\;\text{rate}\left(\frac{\%}{\text{day}}\right)=\frac{\left[(\text{ln}\;\text{final}\;\text{weight}-\text{ln}\;\text{Initial}\;\text{weight})\right]}{\left[\text{Final}\;\text{time}-\text{Initial}\;\text{time}\right]}\times 100$$

$$\text{Feed}\;\text{conversion}\;\text{ratio}\;\text{(FCR)}=\frac{\text{Total}\;\text{feed}\;\text{given}\;\text{(Dry}\;\text{weight)}}{\text{Total}\;\text{weight}\;\text{gain}\;\text{(Wet}\;\text{weight)}}$$

$$\text{Condition}\;\text{factor}\;(\text{K})=\left[\frac{\text{Weight}}{{\text{Length}}^{3}}\right]\times 100$$

$$\text{Hepatosomatic}\;\text{index}\;\text{(HSI)}\;\text{(\%)}=\left[\frac{\text{Weight}\;\text{of}\;\text{liver}}{\text{Total}\;\text{body}\;\text{weight}}\right]\times 100$$

$$\text{Viscerosomatic}\;\text{index}\;(\text{VSI})(\text{\%})=\left[\frac{\text{Visceral}\;\text{weight}}{\text{Total}\;\text{body}\;\text{weight}}\right]\times 100$$

$$\text{Survival}\;\text{rate}\;(\%)=\left[\frac{\text{Number}\;\text{of}\;\text{surviving}\;\text{fish}}{\text{Initial}\;\text{number}\;\text{of}\;\text{fish}}\right]\times 100$$

Blood was collected from caudal vein and stored in pro-coagulation clot activator and EDTA coated tubes, respectively. Clot activator tubes were employed to obtain serum, while EDTA coated tubes were utilized for analysis of hematology and blood biochemistry. Blood samples were centrifuged at 5000 rpm for 20 min to extract plasma. It was stored at -20°C until assayed. Muscle and intestine samples were collected and stored at -20°C to determine chemical composition, profile of amino acids and digestive enzymes.

### 2.4 Chemical composition and amino acid analysis

The chemical composition of body muscles was analyzed using the protocol outlined by the Association of Official Analytical Chemists [42]. Muscle samples were dried in an oven at 80°C until a constant dry weight was achieved. These dried samples were then ground for further chemical analysis. The crude protein was determined using the Kjeldahl apparatus (PCSIR, Pakistan). Crude lipids were determined by following Folch method [43] in the Soxhlet apparatus (PCSIR, Pakistan). The ash content in the muscles were determined by using the furnace burning method. An amino acid analyzer (Biochrome 30+, Biochrome limited, Cambridge, UK) was used to quantify the amino acid contents of fish muscles and the analytical protocols followed by Ahmed et al [44].

### 2.5 Digestive enzymes assay

Crude enzymatic extracts from intestine samples were prepared Ding et al [45]. Properly rinsed intestine samples were homogenized in the phosphate buffer saline (PBS) (pH 7.5) (1 g/10 ml and centrifuged at 5000 rpm for 20 minutes. The resultant supernatant was procured and preserved at 4°C. All analyses were performed within a few hours following the extraction process. Protease activity of intestine samples was determined using Folin-phenol reagent, according to Jin [46]. Quantification of amylase enzymes activity was carried out by utilizing iodine to detect the unhydrolyzed starch in samples, as followed by Jiang [47]. Lipase enzymatic activity was assessed by measuring the fatty acids released through the enzymatic breakdown of triglycerides in a stabilized dispersion of olive oil droplets, as described by Borlongan [48]. The enzymatic activities are expressed as intestine content units per liter (U/L).

### 2.6 Hematology, blood biochemistry and assays of antioxidant biomarkers

The level of red blood cells (μL), mean corpuscle volume (MCV) (fL), haemoglobin (g/dl), mean corpuscular haemoglobin (MCH) (%), haematocrit (HCT) (%), mean corpuscular haemoglobin concentration (MCHC) (%), white blood cells (μL), platelets (μL), eosinophils (μL), neutrophils (μL), monocytes (μL) and lymphocytes (μL), were measured by using clinical hematology analyser (Sysmex, China). Blood glucose level (mg/dl) was measured by using laboratory blood glucose analyser. Cholesterol (mg/dl) and triglycerides (mg/dl) were measured by using ELISA (Biocompare, USA), (Abcam, UK) as per manufacturer’s protocol. Alanine aminotransferase (ALT) (U/L), and aspartate aminotransferase (AST) (U/L) were analysed using kits (Thermo Fisher Scientific, USA) on a clinical chemistry analyser (Thermo Fisher Scientific).

The SOD activity [EC.1.15.1.1], was assessed utilizing the (SOD-1 ELISA Kit- PARS BIOCHEM) (Cat No. PRS-02005 hu), providing a direct and kinetic method for quantifying SOD activity. The extent of inhibition is proportionate to the SOD concentration within a specified range (0.3ng/ml- 10ng/ml). SOD activity was determined by measuring the auto-oxidation rates in the presence and absence of the sample, the results were expressed as μmol/L. The activity of catalase (EC:1.11.1.6) were determined spectrophotometrically (560nm) by using catalase colorimetric activity kit (Thermo Fisher Scientific, USA) (Cat No. EIACATC), as per manufacturer instruction. Malondialdehyde (MDA) (EC No. 202-974-4) concentration was determined using ELISA Kit (Cat No. PRS - 00991hu). MDA level was measured within the range of 0.3nmol/ml- 7nmol/ml at 450nm.

### 2.7 Histological analysis

At the end of bacterial challenge, the intestine, gills, liver, muscles, and kidney were collected from each group (n = 5 of each organ) and placed in sterilized tubes containing 3ml of Bouin’s fluid solution (Solarbio, Beijing, China). Following this, the samples were undergoing standard dehydration procedures and were embedded in paraffin. Sections with a thickness of 5μm were then sliced from each sample and subjected to staining with hematoxylin and eosin [49].

### 2.8 Bacterial challenge

#### 2.8.1 Isolation *Staphylococcus aureus*

*S*. *aureus* was obtained from diseased *Labeo rohita* fish originating from the University diagnostic laboratory, Department of Microbiology, University of Veterinary and Animal Sciences, Lahore Pakistan. A 10-gram portion of the afflicted fish sample was blended with 90 ml of sterile peptone water, generating a 1:10 dilution, to facilitate the enrichment of the target bacterial species. Subsequently, this mixture was incubated at 37°C for 6 hours following Akbar and Anal [50]. From dilutions, 0.5 ml was inoculated on to Mannitol Salt Agar (MSA) and incubated at 37°C for 24 hours. The emergence of colonies exhibiting a yellow hue was indicative of *S*. *aureus* and was subsequently validated through gram staining and coagulase production test. The purified subculture was duly preserved to facilitate subsequent analyses, in accordance Akbar and Anal [50].

### 2.9 Challenge with *S*. *aureus*

After the growth experiment, we challenged the fish with *S*. *aureus* for 15 days (September 15 until September 30). The *S*. *aureus* culture was prepared in 10 ml volume of nutrient broth (HiMedia Ltd., Lahore, Pakistan). Subsequently, the culture was vortexed, and incubated within a shaker incubator for a 24 hour at 37°C. The culture was centrifuged (Micro Prime Centrifuge, Pocklington, UK) at 8000 rpm for 15min at 4^◦^C to get the hard pellet. The obtained pellet underwent several washings, employing sterile phosphate buffer saline (PBS). Following the thorough washing process, the pellet was re-suspended in PBS (pH 7.4). To ascertain the optical density of bacterial suspension, a UV spectrophotometer was utilized to obtained a corresponding concentration of 5×10^5^ CFU/ml. The control group was split into two distinct subgroups: positive control (+ve P0) and negative control (-ve P0). Fish in -ve P0 was given bath with PBS only, whereas the other groups (+ve P0, P1, P2, and P3) (n = 15 for each group) were exposed to *S*. *aureus* (5×10^5^ CFU/ml). Fish were bathed for 2 hours and the bath was repeated after seven days. Throughout the challenge period, all fish in different dietary groups were fed their appropriate diets, except for -ve P0 and +ve P0 fish, were specifically fed a diet with zero probiotics. Fig 1 illustrate step wise process of whole methodology.

**Fig 1:** Step wise process of experimental work performed during the growth experiment and bacterial challenge test.

### 2.10 Statistical analysis

The results were presented as mean ± standard error (S.E). Statistical analysis of the data was performed using one-way analysis of variance (ANOVA) with a significance level set at *P*<0.05 to determine significant differences among groups. Based on the normality (Kolmogorov–Smirnov test) and homogeneity of variances (Levene test), any discrepancies between means were further examined using Duncan Multiple Range Test (DMRT). The parameters which showed significant variance after DMRT test have been mentioned with superscripts for all groups. All the Analyses were conducted using SPSS version 20.

## 3. Results

### 3.1 Growth

A significant difference (*P*<0.05) was observed in all growth parameters among four dietary groups (Table 2). These parameters gradually increased with the increase in the concentration of probiotic. P3 showed the highest value of body weight (398.01±16.97g), SGR (1.61±0.03%), K (1.17±0.01%), HSI (1.49±0.01%), and VSI (2.98±0.01%). Similarly, the best FCR (0.89±0.02%) was also recorded in fish fed with P3 diet.

**Table 2:** Summary of growth parameters in four dietary groups at the end of the growth experiment. Different superscripts across the rows represent the variance between treatments were applied as a result of one-way ANOVA (Duncan multirange test) at *P* < 0.05.

Parameters	P0	P1	P2	P3
TBW (g)	217.73±2.51^a^	228.02±8.43^a^	254.06±5.82^b^	398.01±16.97^c^
TBL (cm)	27.07±0.17^a^	27.73±0.28^a^	28.01±0.28^b^	32.39±0.39 ^c^
SGR (%/day)	0.66± 0.02^a^	0.71±0.01^b^	0.87±0.01^c^	1.61±0.03^d^
FCR	2.55±0.01^d^	2.13±0.02^c^	1.71±0.01^b^	0.89±0.02^a^
K (%)	1.10±0.01^b^	1.07±0.01^a^	1.16±0.01^c^	1.17±0.01^c^
HSI (%)	1.01±0.01^a^	1.32±0.01^c^	1.31±0.01^b^	1.49±0.01 ^d^
VSI (%)	2.98±0.02^a^	3.19±0.04^b^	3.36±0.03^c^	2.98±0.01^a^

P0: 0, P1: 1×10^6^, P2: 1×10^8^ and P3: 1×10^10^ CFU/g of *B*. *subtilis*), TBW- total body weight, TBL- total body length, SGR- specific growth rate, FCR- feed conversion ratio, K- condition factor, HSI-hepatosomatic index, VSI- viscerosomatic index

### 3.2 Chemical composition and amino acid profile of muscles

Chemical composition (moisture content, crude protein, crude fat and crude ash) showed a substantial difference (*P*<0.05) among all dietary groups at the end of the growth experiment (Table 3). The level of crude protein between treatment groups directly correlated with a gradual increase in the concentration of probiotics. The highest concentration of crude protein (23.74±0.24%) was observed in the P3 group. The results showed a significant difference (*P*<0.05) between essential amino acids (EAA) and non- essential amino acids (NEAA) among all treatment groups (Table 4). P0 treatment group had substantially (*P*<0.05) lower concentrations of EAA and NEAA concentrations as compared to other treatments (P0<P1<P2<P3).

**Table 3:** Chemical composition of muscles in different dietary groups at the end of the growth experiment. Different superscripts across the rows represent the significant variance between treatments were applied as a result of one-way ANOVA (Duncan multirange test) at *P* < 0.05.

Parameters	P0	P1	P2	P3
Moisture (%)	70.42±0.93^c^	69.01±0.94^b^	69.02±0.93^b^	68.12±0.85^a^
Crude Protein (%)	16.76±0.19 ^a^	19.25±0.01^b^	20.82±0.22^c^	23.74±0.24^d^
Crude Fat (%)	8.26±0.01^d^	6.26±0.11^b^	6.19±0.02^a^	6.17±0.18^c^
Crude Ash (%)	4.43±0.16 ^ab^	4.05±0.05^a^	4.07±0.05^b^	4.32±0.31^ab^

(P0: 0, P1: 1×10^6^, P2: 1×10^8^ and P3: 1×10^10^ CFU/g of *B*. *subtilis*)

**Table 4:** Determination of essential amino acids (EAA) and non-essential amino acids (NEAA) from muscles of different dietary groups at the end of the growth experiment. Different superscripts across the rows represent the significant variance between treatments were applied as a result of one-way ANOVA (Duncan multirange test) at *P* < 0.05.

Essential Amino Acids (mg/Kg)				
**Amino Acids**	**P0**	**P1**	**P2**	**P3**
Methionine	1.47±0.01^a^	1.63±0.01^b^	1.83±0.01^c^	1.92 ± 0.02^d^
Tryptophan	2.43±0.02^a^	2.47±0.01^b^	3.27±0.01^c^	3.56 ± 0.02^d^
Valine	118.33±0.01^a^	167.91±0.02^b^	223.21±0.01^c^	251.72±0.04^d^
Isoleucine	91.05±0.01^a^	104.79±0.05^b^	145.74±0.01^c^	149.24±0.08^d^
Leucine	3.71±0.01^a^	4.15 ±0.01^b^	4.91±0.01^c^	5.01±0.02^d^
Phenylalanine	4.55±0.03^a^	6.23 ±0.01^b^	6.82±0.04^c^	7.11±0.02^d^
Histidine	0.86±0.02^a^	1.17±0.01^b^	1.25±0.02^c^	1.25 ±0.01^c^
Lysine	29.08±0.01^c^	24.75±0.04^a^	27.72±0.03^b^	32.24±0.01^d^
Arginine	9.05±0.17^a^	9.65±0.01^b^	9.84±0.03^c^	11.04±0.03^d^
Ornithine	72.47±0.06^c^	71.63±0.01^b^	74.22±0.05^d^	54.12±0.03^a^
TEAA	332.97	394.38	498.27	517.21
**Non-essential amino acids (mg/Kg)**				
Cysteine	3.45±0.01^b^	3.14±0.01^a^	4.81±0.02^c^	4.85±0.04^d^
Aspartic Acid	4.66±0.01^b^	4.39±0.04^a^	5.56±0.02^c^	5.65±0.05^d^
Asparagine	13.30±0.03^a^	13.39±0.04^b^	16.73±0.03^c^	17.75±0.06^d^
Serine	3.74±0.01^a^	10.55±0.06^b^	15.66±0.02^c^	19.26±0.03^d^
Glutamine	169.5±0.06^a^	171.41±0.02^d^	173.44±0.04^b^	174.05±0.03^c^
Glycine	0.76±0.01^a^	1.66 ±0.01^b^	3.23±0.01^c^	3.39±0.05^d^
Alanine	163.71±0.05^a^	188.18±0.02^b^	188.72±0.03^c^	189.05±0.03^d^
Proline	44.14±0.06^a^	48.54±0.06^b^	48.81±0.05^c^	49.13±0.05^d^
Tyrosine	2.91±0.01^a^	3.81±0.06^c^	3.73±0.08^b^	4.07±0.01^d^
Threonine	1.46±0.02^a^	2.67±0.02^b^	6.03±0.01^c^	6.15±0.01^d^
TNEAA	406.91	447.74	467.32	473.35

(P0: 0, P1: 1×10^6^, P2: 1×10^8^ and P3: 1×10^10^ CFU/g of *B*. *subtilis*), TEAA- Total essential amino acids; TNEAA-Total non-essential amino acids

### 3.3 Digestive enzymes assay

Dietary supplementation of probiotics substantial (*P*<0.05) increased the levels of amylase lipase and protease in the intestine. The lowest levels of lipase were observed in fish fed with P0 diet. The highest level of digestive enzymes was observed in P3 dietary group at the end of the growth experiment (Table 5).

**Table 5:** Determination of digestive enzymes of intestine samples from different dietary groups at the end of the growth experiment. Different superscripts across the rows represent the significant variance between treatments were applied as a result of one-way ANOVA (Duncan multirange test) at *P* < 0.05.

Treatments				
Parameters	P0	P1	P2	P3
Amylase (Unit/L)	44395.72±2.60^a^	45281.21±1.45^b^	48462.54±0.88^c^	64865.65±2.88^d^
Lipase (Unit/L)	364.32±1.15^c^	79.52±0.57^a^	842.23±1.15^d^	242.43±0.88^b^
Protease (Unit/L)	90.21±1.33^a^	143.32±0.57^b^	162.12±1.45^c^	232.52±0.88^d^

(P0: 0, P1: 1×10^6^, P2: 1×10^8^ and P3: 1×10^10^ CFU/g of *B*. *subtilis*)

### 3.4 Hematology, blood biochemistry and antioxidant enzymes assay

All hematological and biochemical parameters showed substantial difference (*P*<0.05) between the four treatment groups both at the end of the growth experiment and after the bacterial challenge. Hematological parameters also showed a similar pattern between dietary groups, except that glucose gradually decreased with an increase in the probiotic (Table 6). These parameters were found to be lower in +ve P0 group as compared with those noted in -ve P0 group after bacterial challenge. The values of all blood biochemistry parameters increased with a gradual increase in the concentration of probiotic except triglycerides, ALT and AST at end of the growth experiment (Table 7). Similar results were observed at the end of the bacterial challenge. CAT, SOD, and MDA were substantially different (*P*<0.05) among all dietary groups (Table 8). The levels of CAT and SOD increased in response to bacterial challenge in *B*. *subtilis* fed groups. The highest level of CAT (2.55±0.01μmol/L) and SOD (0.54±0.03μmol/L) were observed in P3 group. On the other hand, the concentration of MDA gradually decreased with an increase in the probiotic (+veP0 >P1>P2>P3).

**Table 6:** Hematology from different dietary groups at the end of the growth experiment and after bacterial challenge. Different superscripts across the rows represent the significant variance between treatments were applied as a result of one-way ANOVA (Duncan multirange test) at *P* < 0.05.

**Hematology at the end of growth experiment**					
**Parameters**	**P0**	**P1**	**P2**	**P3**	
Glucose(mg/dL)	89.04±0.57^d^	88.12±0.57^c^	78.42±0.33^b^	76.32±0.57^a^	
Hb (g/dl)	7.62 ± 0.05^a^	10.44±0.05^c^	10.12±0.08^b^	11.25±0.05^d^	
WBC (μL)	5.42±0.05^a^	6.31±0.05^b^	6.83±0.03^c^	7.84±0.05^d^	
RBC (μL)	1.71±0.05^a^	2.61±0.05^b^	3.36±0.08^c^	3.51±0.05^d^	
MCV (fL)	168.54±0.33^a^	177.12±0.33^b^	186.34±0.57^c^	211.34±0.57^d^	
HCT (%)	22.24±0.13^a^	31.43±0.05^c^	31.35±0.05^b^	34.65±0.05^d^	
Platelets(μL)	250.63±0.57^b^	235.12±0.57^a^	311.32±0.57^c^	311.45±0.57^c^	
MCH (%)	48.12±0.57^a^	54.11±0.57^c^	52.62±0.33^b^	59.11±0.57^d^	
**Hematology at the end of bacterial challenge**					
**Parameters**	**-ve P0**	**+ve P0**	**P1**	**P2**	**P3**
Glucose(mg/dL)	89.13±0.33^b^	95.52±2.84^d^	91.43±0.33^c^	89.56±0.57^b^	86.72±0.33^a^
Hb (g/dl)	7.45±0.03^b^	6.46±0.03^a^	7.71± 0.05^c^	7.82±0.05^c^	9.44±0.05^d^
WBC (μL)	4.84±0.03^b^	4.13±0.03^a^	5.22±0.05^c^	5.41±0.03^d^	6.82±0.05^e^
RBC (μL)	1.61±0.05^a^	1.21±0.05^a^	1.63±0.03^a^	2.16±0.03^b^	2.51±0.05^c^
MCV (fL)	167.52±0.57^b^	155.54±0.57^a^	173.12±0.57^c^	174.23±0.05^d^	179.34±0.57^e^
HCT (%)	21.84±0.08^b^	19.84±0.08^a^	21.92±0.03^b^	23.83±0.05^c^	28.62±0.03^d^
Platelets(μL)	231.16±0.88^b^	159.62±0.57^a^	275.12±0.57^c^	281.54±0.57^d^	288.63±0.33^e^
MCH (%)	44.72± 0.33^b^	34.33±0.33^a^	44.14±0.57^b^	50.16±0.57^c^	54.15±0.57^d^

-ve P0: negative control (not exposed with S. aureus bacteria), +ve P0: positive control (exposed with S. aureus bacteria), P0: 0, P1: 1×10^6^, P2: 1×10^8^, P3: 1×10^10^CFU/g of the *B*. *Subtilis*, Hemoglobin (Hb), white blood cells (WBC), red blood cells (RBC), mean corpuscle volume (MCV), haematocrit (HCT), mean corpuscular haemoglobin (MCH), μL–microliter, fL- femtoliter

**Table 7:** Blood biochemistry of different dietary groups at the end of the growth experiment and after bacterial challenge. Different superscripts across the rows represent the significant variance between treatments were applied as a result of one way (Duncan multirange test) at *P* < 0.05.

**Blood biochemistry at the end of growth experiment**					
**Parameters**	**P0**	**P1**	**P2**	**P3**	
Neutrophils (μ/L)	19.01±0.57^a^	25.10±0.33^b^	29.21±0.33^c^	35.22±0.57^d^	
Lymphocytes (μ/L)	70.12±0.57^a^	73.12±0.57^b^	76.21±0.33^c^	84.23±1.21^d^	
Monocytes (μ/L)	2.34±0.33^a^	2.01±0.41^a^	5.23±0.33^b^	5.12±0.33^b^	
Eosinophils (μ/L)	2.31±0.33^a^	2.23±0.33^a^	3.12±0.33^b^	4.23±0.33^b^	
Triglycerides(mg/dl)	398.43±0.57^d^	362.12±1.45^c^	359.21±2.61^b^	281.09±1.85^a^	
ALT (Unit/L)	41.72±0.88^d^	35.34±0.57^c^	28.54±0.88^b^	23.56±0.57^a^	
AST (Unit/L)	40.23±0.57^d^	24.12±0.57^b^	19.14±0.57^a^	26.06±0.33^c^	
Total Protein (g/dl)	3.61±0.07^a^	4.41 ±0.08^b^	4.72 ±0.05^c^	4.84 ±0.08^d^	
**Blood biochemistry at the end of bacterial challenge**					
**Parameters**	**-ve P0**	**+ve P0**	**P1**	**P2**	**P3**
Neutrophils (μ/L)	19.21±0.33^b^	16.26±0.33^a^	21.43±0.57^c^	22.54±0.33^c^	24.44±0.33^d^
Lymphocytes (μ/L)	63.32±0.88^b^	60.12±0.57^a^	64.04±0.57^c^	65.52±0.57^c^	70.12±0.57^d^
Monocytes (μ/L)	2.45±0.33^b^	1.72±0.05^a^	2.23±0.33^b^	2.54±0.33^b^	4.62±0.57^c^
Eosinophils (μ/L)	2.72±0.05^a^	2.12±0.05^a^	2.12±0.06^b^	2.62±0.33^a^	3.12±0.33^c^
Triglycerides(mg/dl)	397.12±1.15^d^	399.45±5.78^e^	384.12±2.61^c^	374.21±2.3^b^	364.43±2.08^a^
ALT (Unit/L)	44.32±0.33^c^	51.12±1.85^d^	39.24±0.57^b^	37.02±0.88^a^	37.42±0.88 ^a^
AST (Unit/L)	41.45±0.33^d^	46.25±0.57^e^	40.24±0.57^c^	37.52±1.21^b^	35.41±1.21^a^
Total Protein (g/dl)	3.62±0.05^c^	2.71±0.08^a^	3.33±0.05^b^	3.64±0.03^c^	3.86±0.05^d^

-ve P0: negative control (not exposed with S. aureus bacteria), +ve P0: positive control (exposed with S. aureus bacteria), P0: 0, P1: 1×10^6^, P2: 1×10^8^, P3: 1×10^10^CFU/g of the *B*. *Subtilis*, alanine aminotransferase (ALT), aspartate aminotransferase (AST), μ/L- micro liter

**Table 8:** Determination of catalase (CAT), malondialdehyde (MDA) and superoxide dismutase (SOD) from serum of different dietary groups at the end of the growth experiment and after bacterial challenge. Different superscripts across the rows represent the variance between treatments were applied as a result of one way (Duncan multirange test) at *P* < 0.05.

**At the end of the growth experiment**					
**Parameters**	**P0**	**P1**	**P2**	**P3**	
Catalase (μmol/L)	0.50±0.01^a^	0.54±0.01^b^	0.54±0.01^b^	0.63±0.01^c^	
MDA (μmol/L)	0.41±0.01^d^	0.34±0.01^c^	0.28±0.01^b^	0.24±0.01^a^	
SOD (μmol/L)	0.20±0.04^a^	0.33±0.01^b^	0.36±0.01^b^	0.39±0.01^c^	
**At the end of the bacterial challenge**					
**Parameters**	**-ve P0**	**+ve P0**	**P1**	**P2**	**P3**
Catalase (μmol/L)	1.51±0.02^b^	0.15±0.01^a^	1.70±0.01^c^	2.31±0.06^d^	2.55±0.01^e^
MDA (μmol/L)	0.33±0.01^d^	0.35±0.01^e^	0.31±0.01^c^	0.24±0.01^b^	0.20±0.03^a^
SOD (μmol/L)	0.47±0.01^d^	0.31±0.01^a^	0.42±0.01^b^	0.44±0.01^c^	0.54±0.03^e^
Survival Rate (%)	100	40	90	100	100

-ve P0: negative control (not exposed with S. aureus bacteria), +ve P0: positive control (exposed with *S*. *aureus* bacteria), P0: 0, P1: 1×10^6^, P2: 1×10^8^, P3: 1×10^10^CFU/g of the *B*. *Subtilis*, μmol/L: micro moles per liter

### 3.5 Histological study

The gut structure of different treatment groups showed several pathologies (Fig 2A–2E). Histopathological analysis of the -ve P0 showed a normal or less alterations of goblet cells, villi, and nuclei (Fig 2A). Meanwhile, the other treatment groups revealed structural anomalies such as excessive hypertrophy, the villi tended to fuse (FV), and the mucosal lining sloughed off, eventually leading to the large lumen (LL) (Fig 2B–2E).

**Fig 2:** Histological changes in gut. Light micrographs of a paraffin section stained with eosin (40x). a; gut in -veP0, b; gut in P1, c; gut in P2, d; gut in P3, e; gut in +ve P0. GC; Goblet cells, LP; Laminar propria, N; Nucleus, L; Lumen, CE; Columnar epithelium, FV; Fusion of villi, LL; Large lumen, FLV; Flattened villi, DCML; Damaged circular muscle layer, DL; Distended lumen, DLML; Damaged longitudinal muscle layer, VF; Vacuole formation, SLP; Swelling of lamina propria, CCA; Cracked clay appearance of the tissues, SLML; Swelling of longitudinal muscle layer, DGC; Damaged goblet cells, DMM; Disarrangement of muscularis mucosa.

Several histopathological alterations were observed in the structure of gills in all treatment groups (Fig 3A–3E). The histology of gills in the -ve P0 group exhibited the typical epithelial cell lining of lamellae (Fig 3A). In contrast, the groups exposed to *S*. *aureus* showed various structural changes, such as hemorrhage, intracellular oedema, disruption of gills with notable hypertrophy, loss of horizontal shaft with mucous membrane cellular proliferation (Fig 3B–3E). Liver in different treatment groups showed significant abnormalities (Fig 3F–3J). The group fed with zero probiotic (-ve P0) revealed normal hepatocytes, endothelium and serous membrane that contained blood vessels (Fig 3F). On the other hand, treatment groups showed pathologies such as necrosis, multinucleated nucleolus, oedema, hemosiderin, hematoma, intravenous tissue necrosis, edematous fluid intrusions (Fig 3G–3J).

**Fig 3:** Histological changes in gills and liver. Light micrographs of a paraffin section stained with eosin (40x). a; gills in -veP0, b; gills in P1, c; gills in P2, d; gills in P3, e; gills in +veP0, f; liver in -veP0, g; liver in P1, h; liver in P2, i; liver in P3, j; liver in +veP0. PL; Primary lamellae, SL; Secondary lamellae, FSL; Fusion of secondary lamellae, DSL; Degeneration of secondary lamellae, HT; Hypertrophy, DPL; Degeneration of primary lamellae, TD; Tissue debris, A; Aneurism, H; Hypertrophy, NH; Normal hepatocytes, GC; Granular cytoplasm, BC; Blood congestion HD; Hepatocyte generation, CSN; Central spheroidal hepatocyte nucleus, N; Cell necrosis, PN; Pyknotic nuclei, CD; Cytoplasmic degeneration, IEF; Infiltration of oedematous fluid, rCV; Rupturing of the central vein, V; Vacuolization of hepatocytes.

Several anomalies were observed in the muscle’s structures of different treatment groups after bacterial challenge (Fig 4A–4E). Muscle structures of the -ve P0 group showed less or no abnormalities (Fig 4A) as compared to other treatment groups. Whereas, different treatment groups showed notable structural changes including, muscle fibers degeneration, vacuole destabilisation in muscle bundles and the increased inter myofibrillar space (IMFS) (Fig 4B–4D). The highest pathological alterations were observed in muscles of the +ve P0 group (Fig 4E). The kidney structure of different treatment groups exhibited anomalies (Fig 4F–4J). Less or no structural abnormalities were observed in kidney structure of -ve P0 group (Fig 4F). However, the +ve P0 group displayed the highest structural abnormalities among all other treatment groups (Fig 4J). Severe structural changes among treatment groups were observed (P1>P2>P3) (Fig 4G–4I).

**Fig 4:** Histological changes in muscles and kidney. Light micrographs of a paraffin section stained with eosin (40x). a; muscles in -ve P0, b; muscles in P1, c; muscles in P2, d; muscles in P3, e; muscles in +veP0, f; kidney in -ve P0, g; kidney in P1, h; kidney in P2, i; kidney in P3, j; kidney in +ve P0. MF; Myofibrils; GFMF; Gap formation in myofibril, IMFS; Inter myofibrillar space, DMF; Disintegrated myofibrils, EMF; Oedema between muscle fibre, MD; Muscle degradation, ME; Muscle oedema, G; Glomerulus, CD; Collecting duct, DG; Degenerative glomerulus, IBS; Increased bowman space, FRT; Fusion of renal tubule, DRT; Degenerative renal tubule, CG; Congestion of glomerulus, N; Necrosis, H; Hemorrhage, A; Atrophy.

## 4. Discussion

The present study demonstrated a significant increase in various growth parameters, such as total body weight (%), SGR (%), K (%), and HSI (%) after feeding fish with different doses of *Bacillus subtilis*. The condition factor is closely linked to the weight–length ratio [51], reflecting fish’s physiological and biological state. The fluctuations in the condition factor depends upon the feeding conditions, disease prevalence, and physiological factors [52]. Condition factor in all probiotic fed groups indicate that the inclusion of *B*. *subtilis* ensured favorable health conditions and isometric growth throughout the growth period. Similar positive outcomes were observed in tilapia when administered with bacillus probiotic [21].

The findings of this study presented conclusive evidence that the substantial increase in weight gain resulting from probiotic supplementations can be attributed to an increased digestive enzyme functioning in striped catfish. The gastrointestinal enzymes were significantly increased in the treatment groups. These results are consistent with previous studies on freshwater species such as Nile tilapia [53], grass carp, and African catfish [54], *B*. *subtilis* possesses the capacity to improve the breakdown of nutrients in the gut, resulting in increased energy availability for fish growth. Previous studies have demonstrated that probiotics can generate a diverse array of exo-enzymes and enhance the functioning of the digestive enzymes within the gut [55]. Furthermore, the inclusion of dietary probiotics can have an impact on the composition of the intestinal microbiota in fish. As a result, their administration can lead to the proliferation of advantageous microorganisms in the gut, ultimately enhancing the functioning of digestive [56].

Other than elevation in digestive enzymes, the present study revealed that striped catfish had enhanced crude protein content (23.74±0.24%), which consequently led to an augmentation in muscle protein. The elevated protein content implies that incorporating probiotics in the feed resulted in a more effective conversion of nutrients into structural proteins, ultimately leading to better muscle production [57]. The result coincides with findings in Nile tilapia and rainbow trout [58, 59]. An increase in body protein body protein levels demonstrated a significant rise in both dispensable and indispensable amino acids, particularly in P3 group. This study identified valine as an abundant amino acid, which had crucial role in cellular regeneration, muscle growth, and development. Furthermore, it serves as precursor in the production of antimicrobial agents. Dispensable amino acids showed significant increase in different treatment groups. These amino acids are essential for efficient utilization of essential amino acids and synthesis of various biological nitrogen containing molecules, including pyrimidines and purines, as well as antioxidant enzymes like glutathione [60].

The present study demonstrated that the utilization of *B*. *subtilis* resulted in a significant enhancement of hematological parameters specifically in the counts of RBC and WBC. These cells play a crucial role in the circulation of oxygen within the respiratory system and blood flow regulation [61], as well in innate and adaptive immunity [62]. Previous studies have demonstrated that probiotics containing a mixture of bacillus strains can improve the haematological profiles of *O*. *niloticus* [21, 63] and rainbow trout [64]. The +ve P0 group exhibited the highest glucose level compared to other treatments after bacterial challenge, indicating the increased tissue requirements to fuel the metabolic needs of osmoregulation and serves as the vital energy source for maintaining homeostasis [65] as well as assist fish in adapting to constant changes in metabolic demands [66].

Meanwhile, the current study demonstrated that the treatment groups supplemented with probiotics exhibited a significant improvement in the antioxidant response, as indicated by biomarkers (SOD, CAT and MDA). These results suggest that *B*. *subtilis* can stimulate the secretion of antioxidant enzymes in striped catfish, thereby enhancing the immune response, as observed in several other species [33, 67]. The SOD and CAT activities were observed to be lowest in the +ve P0 and -ve P0 groups, indicating a weakening of antioxidant defense, which could potentially lead to tissue damage caused by excessive free radicals. The persistence of free radicals can have detrimental effects on the normal functioning of cells. The excessive buildup of reactive oxygen species (ROS) can disrupt cellular metabolism and potentially lead to cell death [68].

Reactive oxygen species, which include superoxide radical, hydroxide anion and peroxide (H_2_O_2_), are generated during cellular phagocytosis and catabolism processes. To counteract the harmful effects of ROS, key biochemical factors i.e., superoxide dismutase, glutathione and catalase act as the body’s first line of defense. These parameters modulate the presence of oxidative radicals and protect the body against oxidative pressure [69]. Present results showed that *S*. *aureus* infection led to a significant augmentation in MDA levels in the +ve P0 group, which indicates damage in DNA, protein and cytoplasm. The redox imbalance resulting from lipid peroxidation by a microbe or an additive directly relates to MDA level [32]. Whereas MDA level declined in groups fed diets containing *B*. *subtilis* and subsequently exposed to bacterial challenge. This decline could signify the presence of enzymatic regulators and non-enzymatic free radical quenchers that counteract the detrimental effects of ROS and reduce the rate of fatty acid peroxidation [18]. The histological alterations during the bacterial challenge test correlated with haemato-biochemical and antioxidant enzyme data. This study elucidates notable variations in the various tissues, including muscles, gills, kidneys, liver, and gut. The greatest tissue damage was observed in the +ve P0 group. Histopathology, which is the study of tissue damage, is used to examine the effects of various chemicals or infections of biological origin [70, 71]. The gills, due to their perpetual exposure to the external environment, are particularly susceptible to waterborne pathogens [72, 73]. In +ve P0 group, the gills displayed a significant prevalence of histological abnormalities when compared to treatment groups. This result in erythrocytes congestion within the marginal channel [74]. In contrast, the liver histology of probiotic treated groups showed characteristics reminiscent of those found in negative control group (-ve P0). The liver’s impaired ability to efficiently remove foreign particles results in the degeneration of hepatocytes and congestion within sinusoid’s [75]. The presence of extracellular toxin generated by *S*. *aureus* might be the underlying factor responsible for the formation of lipid vacuoles and the occurrence of necrosis in the liver [76, 77]. Comparable hepatic irregularities, including the infiltration of lymphocytes, focal necrosis and the presence of cytoplasmic fat vacuoles, have been similarly observed in various species, such as carp [78]. In fish exposed with *S*. *aureus*, the kidney tissues displayed severe necrosis and observable changes in the glomeruli. Notably, the glomerular epithelium in the kidney of catfish afflicted by *S*. *aureus* exhibited noticeable histological alterations [79]. A pronounced elevation in the height of intestinal villi and reduction in adverse effects of *S*. *aureus* within the probiotic groups might be due to action of *B*. *subtilis* inhabiting the intestine, cause consequent reduction in pH and inhibit fermenting indigestible carbohydrates. Comparable investigation conducted [80] by supplementation of lactobacillus probiotic. Histopathological results support and confirm our examined hematological parameters and consistent with previous findings of pathological examination of *S*. *aureus*.

## 5. Conclusions

In conclusion, the present investigation exhibited that supplementation of *B*. *subtilis* could serves as optimal probiotic concerning growth performance, protein content, antioxidant response and immunocompetency against *S*. *aureus* in striped catfish. The optimum dosage of *B*. *subtilis*, at a concentration of 1×10^10^ CFU/g, resulted in the most favorable outcomes in striped catfish. Moreover, the prospective utilization of *B*. *subtilis* presents a favorable opportunity to replace antibiotics in the context of aquaculture production. Further, the results of this study could suggest that this single bacterial strain probiotics have the potential for intensive farming to improve growth and immune responses in catfish farms, and effective probiotic in large scale production of aquafeed for striped catfish.

## Supporting information

S1 Data (XLSX)
